# Surgical Adhesive Drape (IO-ban) as Postoperative Surgical Site Dressing

**DOI:** 10.7759/cureus.394

**Published:** 2015-12-04

**Authors:** Daniel Felbaum, Hasan R Syed, Rita Snyder, Jason E McGowan, Ribhu T Jha, Mani N Nair

**Affiliations:** 1 Neurosurgery, Medstar Georgetown University Hospital

**Keywords:** spine infection, surgical site infections, postoperative infection

## Abstract

Study Design: Retrospective chart analysis.

Objective: The objective of this study is to describe the senior author’s (MNN) experience applying a widely available surgical drape as a postoperative sterile surgical site dressing for both cranial and spinal procedures.

Summary of Background Data: Surgical site infection (SSI) is an important complication of spine surgery that can result in significant morbidity. There is wide variation in wound care management in practice, including dressing type. Given the known bactericidal properties of the surgical drape, there may be a benefit of continuing its use immediately postoperatively.

Methods: All of the senior author’s cases from September 2014 through September 2015 were reviewed. These were contrasted to the previous year prior to the institution of a sterile surgical drape as a postoperative dressing.

Results: Only one surgical case out of 157 operative interventions (35 cranial, 124 spinal) required operative debridement due to infection. From September 2013 to September 2014, prior to the institution of a sterile surgical drape as dressing, the author had five infections out of 143 operations (46 cranial, 97 spinal) requiring intervention.

Conclusion: The implementation of a sterile surgical drape as a closed postoperative surgical site dressing has led to a decrease in surgical site infections. The technique is simple and widely available, and should be considered for use to diminish surgical site infections.

## Introduction

Postoperative surgical site infections (SSI) can be associated with a considerable amount of health care costs, resources, and patient morbidity [1]. There have been numerous studies that have identified either patient-related or surgeon-related risk factors that can affect postoperative SSI. Patients with advanced age, diabetes, history of smoking, and underlying etiology, such as trauma, elevated body mass index (BMI), large operative blood volume loss, prolonged operative time, and involvement of trainees, have been noted to have a higher rate of infections [2-10]. On the other hand, adhering to scheduled administration of prophylactic antibiotics with appropriate weight-based dosage has been shown to significantly decrease postoperative SSI [2-3]. Topics less thoroughly reviewed include the type of skin preparation, use of a postoperative drain, or wound dressing management in the postoperative period [11-17]. 

The IO-ban surgical drape has been around for thirty years, and its use has been shown to decrease SSI [18-19]. In addition to its bactericidal properties, the drape prolongs sterility by acting as a sterile adhesive around the surgically prepped site [20]. Using larger databases, general surgery literature has compared the efficacy of various skin preparations, such as Dura Prep, Chlora Prep, or iodine-based skin washes. In some studies, the use of IO-ban has aided in decreasing contamination of the surgical field [21]. Inherently, it may decrease postoperative infections by decreasing the amount of bacteria that may become impregnated during surgery [18]. This has been retrospectively reported in neurosurgical literature for intracranial shunting procedures [22]. There is in vitro literature reporting at 30, 60, and 90 minutes of exposure in which the IO-ban drape significantly reduced microbial counts, including MRSA and MRSE [11, 23]. We attempt to review a single surgeon’s experience in instituting a sterile surgical adhesive drape, IO-ban, as a postoperative dressing and surgical site infection.

## Technical report

### Methods

A retrospective analysis was performed prior to and subsequent to the adaptation of a sterile surgical adhesive drape for postoperative dressing. Prior to the institution, the senior author performed 143 operations (46 cranial, 97 spinal), of which five required operative debridement due to surgical site infection. After institution of sterile adhesive drape, only one case required surgical intervention for infection out of 157 operations (35 cranial, 124 spinal). The one surgical case involved a 78-year-old female with diabetes and metastatic breast cancer requiring intradural surgery with spinal instrumentation from L2 to S1. The cultures were positive for Serratia. The patient was treated with prolonged antibiotics (meropenem) without removal of the spinal hardware. The results of patients requiring operative debridement are summarized in Table 1.

**Table 1:** List of patients that underwent surgical debridement Abbreviations: *: IO-Ban Use, PSF - posterior spinal fusion, MRSA - methicillin-resistant Staphylococcus aureus, BMI: body mass index, DM: diabetes mellitus, CAD: coronary artery disease, HTN: hypertension

Patient Profile				
Age	Location	Treatment	Infection	Co-morbidity
60	Spinal (L2-5 PSF)	Wound debridement, IV antibiotics	MRSA	Morbid obesity (BMI>35), >1L intraop blood loss
63	Spinal with hardware (T10 to Iliac PSF)	Multiple wound/spinal revisions, IV antibiotics	MRSA	DM, steroid-dependent COPD, CKD
89	Spinal (L2-5 PSF)	IV antibiotics	MRSA	CAD, poorly controlled HTN, poor nutrition
53	Cranial (L1-4 PSF)	Wound debridement, IV antibiotics	MRSA	Cancer, poorly controlled HTN
52	Spinal (L4-5 PSF, separate surgery hardware revision)	IV antibiotics	MRSA	Morbid obesity, HTN,
73*	Spinal L2-S1 PSF	Wound debridement, Abx	Serratia	Cancer, poor nutrition

### Technique

The wound is copiously irrigated with an antibiotic solution at the conclusion of the operation. The deep fascial layer is closed with 0-Vicryl sutures in an interrupted fashion, followed by the submucosal layer with 2-0 Vicryl sutures in a similar manner. Upon completion, the subcutaneous layer is closed with a running 3-0 Plus Monocryl suture (Ethicon, California). The wound is then covered with Dermabond (Ethicon, California), Telfa non-adherent dressing (Covidien, Dublin, Ireland). Then, using IO-ban surgical adhesive tape (3M, Canada), the wound is covered in a closed manner. The surgical adhesive tape is maintained on the incision during the hospital stay, in an attempt to promote sterility and the bactericidal effects of the dressing. During removal of the surgical drain, the minimum amount necessary is removed, while the remainder of the dressing is maintained during the hospital stay. Antibiotic prophylaxis is maintained during the duration of the drain placement. Appropriate weight-based dosing of Cefazolin or Vancomycin for penicillin-allergic patients is generally used for at least 48 hours.

### Results

A 0.64% (one out of 157) incidence of postoperative infection was noted after implementing the sterile post-surgical adhesive dressing. Prior to that, five out of 143 surgical cases resulted in an overall 3.5 % incidence of infection. A Fisher t-test analysis was performed that did not reveal significance between the two groups (p=.10), although there was a trend to decreased infections in the IO-ban group. This statistical test was elected due to the small population size and in order to compare whether the use of IO-ban affected infection rates.

## Discussion

There has been a multitude of research performed regarding postoperative infections for spinal surgery [2-10]. In other neurosurgical literature, limiting the number of assistants and wearing two sets of gloves have been shown to decrease infections as well [14]. More inherent to the operation, the amount of blood loss, the length and levels of surgery, and underlying etiology of the surgical procedure (trauma or oncologic) have also been associated with an increased risk for postoperative infections [1-2, 15]. In an effort to decrease methicillin-resistant staph aureus (MRSA) infections, the use of a Chloraseptic wash preoperatively has also been employed [16]. Recently, the application of vancomycin powder has been used in spinal procedures and may be associated with decreasing postoperative infection [1].

The postoperative wound care science appears to fall more into the realm of myth, with little-reported data regarding dressing care, time allotted for patient bathing, and postoperative drain use [9]. At the baseline comparative year in this study, antibiotics were continued while drains were in place, although there is no data to support this practice [6]. In addition, routine wound management, for both cranial and spinal patients, involved removal of the closed surgical dressing on postoperative day #2, and allowed for bathing or cleansing on postoperative day #3. Wound dressings were not routinely replaced after the initial removal. Although not used initially, an antibiotic-impregnated suture is commercially available for use, such as Monocryl Plus (Ethicon). In vitro studies have shown the decreased colonization of the suture line between three to five days after surgery, as compared to non-antibiotic impregnated suture [24-26]. This may allow an improved sterile setting for wound epithelization and granulation tissue to the surgical site. The improved surgical site infection rates have been validated in general surgery studies [27]. In addition to the sterile IO-ban dressing, Dermabond (Ethicon) was included in the wound closure. Dermabond alone has been shown to have topical antimicrobial barrier properties as well [27]. Together with meticulous attention to sterile technique, the addition of an antibiotic impregnated suture in combination with a protective wound barrier with prolonged application of IO-ban dressing may provide a synergistic effect in providing the most sterile environment for the initial wound healing. A potential criticism for these multiple mechanisms to prevent infection is that bacterial drug resistance may result if an infection occurred. 

Although the current study did not reveal a statistically significant effect in postoperative surgical site re-operations, the study was not designed to review potential local infections that may have been treated with oral antibiotics and local wound care. This may be a potential future inclusion in another study. There was a trend towards significance in the IO-ban group, which may become statistically significant in a larger surgical cohort over a prolonged period of time, and is currently being reviewed in our institution. In addition, the re-operation rate for infection was low in both groups, which would need a larger cohort for comparison to allow for statistical significance. There are many limitations to this study, including it being a retrospective single surgeon experience, allowing for a potential reviewer bias. In addition, there were several new variables implemented during the study, including the routine use of Dermabond, which may have had an effect on infection rate. A prospective study controlling for the multiple variables affecting surgical site infection would be best for providing information regarding postoperative wound management.

## Conclusions

The implementation of a new prolonged closed sterile postoperative adhesive dressing did not statistically have a lower rate of infection, but there was a trend towards decreased surgical debridement for cranial and spinal surgeries. The use of closed sterile dressing, antibiotic impregnated suture, and an additional wound barrier seal may provide the most conducive environment for decreasing SSI, although further studies are warranted.
